The article "miR-28-5p's Targeting of GAGE12I Inhibits Proliferation, Migration, and Invasion of Gastric Cancer in Vitro" was retracted in 2023. Reasons: unreliable results or conclusions; concerns about the data; concerns about the peer review; concerns about the citations.

# miR-28-5p's Targeting of GAGE12I Inhibits Proliferation, Migration, and Invasion of Gastric Cancer in Vitro

**DOI:** 10.1155/2022/6946051

**Published:** 2022-09-30

**Authors:** Ruizhe Xu, Qi Guo, Peifeng Zhao, Haiyan Lu, Bo Zhang

**Affiliations:** ^1^Department of Radiotherapy & Oncology, The Second Affiliated Hospital of Soochow University, Suzhou, China; ^2^Institute of Radiation Oncology, Soochow University, Suzhou, China

## Abstract

GAGE12I is a tumor metastasis-promoting factor, which can induce gastric cancer cells to invade and migrate. We investigated the effect of miR-28-5p targeting GAGE12I on proliferation, invasion, and migration of human gastric cancer cell lines SGC-7901, AGS, and MGC-803. The expression levels of miR-28-5p and GAGE12I were detected by real-time PCR and western blot, respectively. Cell proliferation, migration, and invasion were measured by MTT and Transwell chamber. The interaction between miR-28-5p and GAGE12I was investigated by bioinformatics analysis and luciferase assay. Results showed that the expression of miR-28-5p in human gastric cancer cell lines was lower than that in normal gastric epithelial cells (*P* < 0.05). Overexpression of miR-28-5p suppressed cell proliferation, invasion, and migration (*P* < 0.05). GAGE12I was confirmed as a target of miR-28-5p. Cell proliferation, invasion, and migration were decreased in cells transfected with shGAGE12I compared with those of the scrambled group (*P* < 0.05). Collectively, miR-28-5p negatively regulated GAGE12I and reduced the proliferation, invasion, and migration of gastric cancer cells.

## 1. Introduction

Gastric cancer is one of the most common malignant tumors, with very complicated pathogenesis. Metastasis of gastric cancer is an important cause of death. The invasion and migration of gastric cancer cells are regulated by a variety of genes. It is important to study the molecular pathogenesis of gastric cancer cells for the treatment of cancer [1]. MicroRNAs (miRNAs) are a class of highly conserved single-stranded RNA, which can induce or inhibit the translation of mRNA by binding to the target gene's mRNA molecules [2]. miR-28-5p is one of the miRNAs existing in human tissues, which is involved in the occurrence of tumors. It has been found that the expression of this miRNA in renal and colon cancer is downregulated, suggesting that miR-28-5p may play an inhibitory role in tumors [3, 4]. However, the role and mechanism of miR-28-5p in gastric cancer remain largely unknown. GAGE12I is a tumor metastasis-promoting factor, which can induce gastric cancer cells to invade and migrate [5]. In this study, we investigated the expression level of miR-28-5p in gastric cancer cells, and studied the effect and mechanism of miR-28-5p on proliferation, invasion, and migration of gastric cancer cells, in order to provide a reference for clarifying the mechanism of gastric cancer progression.

## 2. Materials and Methods

### 2.1. Material

Human gastric cancer cell lines SGC-7901, AGS, and MGC-803 [6] were purchased from Shanghai Cell Bank of the Chinese Academy of Sciences; normal gastric epithelial cells GES-1 was purchased from ATCC of USA; a reverse transcription kit was purchased from Thermo Fisher of USA; GAGE12I antibody was purchased from Abcam of USA; SYBR Green real-time PCR kit was purchased from Shanghai Saobao Biotechnology; miR-28-5p mimics and mimics control was purchased from Balmico Biotechnology; and GAGE12I shRNA and shRNA control from Beijing Ao Rui Dongyuan Biotechnology. All experiments were done in triplicates.

### 2.2. Real-Time PCR Assay

Trizol reagent was added to human gastric cancer cell lines SGC-7901, AGS, and MGC-803 and normal gastric mucosal epithelial cells GES-1 for RNA extraction. RNA was stored in a refrigerator at −80°C. The reverse transcription kit was used to get cDNA. The primers for RT-PCR reaction were: miR-28-5p forward primer: 5′-GCG CAT TGC ACT TGT CTC G-3′, reverse primer: 5′-AGT GCA GGG TCC GAG GTA TT-3′. The U6 was used as control (forward primer: 5′-CTC GCT TCG GCA GCA CATA-3′, reverse primer: 5′-CGA ATT TGC GTG TCA TCCT-3′). The PCR reaction consisted of a 2 × SYBR Green mix of 10 *μ*L, RT product of 2 *μ*L, forward primer and reverse primer of 0.8 *μ*L each, and ddH_2_O of 6.4 *μ*L. The real-time quantitative PCR was performed with the CFX96 real-time PCR instrument (Bio-Rad, USA). The PCR program was: 95°C 20 s, 95°C 10 s, 60°C 20 s, and 72°C 10 s, with a total circulation of 40 times. The quantification was done using the comparative Ct (2^−ΔΔCt^) method.

### 2.3. Cell Transfection

SGC-7901 cells were seeded into 6 well plates, each containing 5 × 10^5^ cells, and incubated at 37°C under 5% CO_2_ overnight. When cell density was 50%, cell transfection was performed. miR-28-5p mimics, mimics control, GAGE12I shRNA, or shRNA control were added to Opti-MEM containing 245 *μ*L and incubated at room temperature for 20 minutes. Opti-MEM was incubated at 37°C for 4 hours. Opti-MEM was removed and cells were washed twice with PBS. RPMI1640 medium containing 10% FBS was added and incubated at 37°C for 48 hours. The SGC-7901 cells transfected with miR-28-5p mimics, mimics control, GAGE12I shRNA, or shRNA control were recorded as miR-28-5p, miR-NC, shGAGE12I, or scrambled group, respectively.

### 2.4. MTT Assay

miR-28-5p and miR-NC groups cells were inoculated into a 96-well plate at a concentration of 6 × 10^4^/mL in 100 *μ*L cell culture medium per well and incubated for 24 h, 48 h, or 72 h. Methylthiazolyl diphenyl-tetrazolium bromide (MTT) solution of 10 *μ*L was added into each hole and cells were incubated at 37°C for an extra 4 h. The supernatant solution in the well was absorbed, and 150 *μ*L dimethyl sulfoxide (DMSO) solution was added. The supernatant was shaken in a low-speed shaker for 10 min. OD value at 570 nm was measured for enzyme-linked immunosorbent assay (ELISA). Cell viability was calculated according to the manufacturer's manual [7].

### 2.5. Transwell Chamber Assay

Invasion experiment: Matrigel was dissolved at 4°C, and the RPMI1640 medium was preheated at 4°C and diluted with Matrigel. Then the residual liquid was collected out of the well. miR-28-5p and miR-NC groups cells were inoculated into the well compartment and 5 × 10^4^ cells were added to each well. After incubation for 24 hours, the cells that had not penetrated the membrane were wiped off and the number of invasive cells was counted under a 200-fold microscope.

### 2.6. Prediction and Identification of Target Genes

According to the bioinformatics analysis by TargetScan and Pitar software, the target gene of miR-28-5p may be GAGE12I. Wild-type (WT) and mutant-type (MUT) luciferase reporter vectors were constructed according to GAGE12I 3-UTR binding sites and were cotransfected into SGC-7901 cells with miR-28-5p mimics, or mimics control, respectively, then detected by measurement of luciferase activity.

### 2.7. Western Blot

miR-28-5p and miR-NC groups cells were collected with the addition of RIPA buffer (Thermo Fisher, USA). The cells were lysed on ice for 1 h and centrifuged at 4°C for 15 minutes. The concentration of the supernatant of cell lysate was measured using the BCA kit (Thermo Fisher, USA). Each lysate sample containing 30 *μ*g protein was mixed with SDS loading buffer and boiled for 10 minutes, followed by loading onto a 5% concentrating +12% separating gel. The initial voltage was 80 V at the concentrating gel and then adjusted to 120 V when the samples entered the separating gel. The electrophoresis was continued for about 1 h, and the proteins were transferred onto a PVDF at 100 V voltage for 1 h. The PVDF membrane was incubated in 5% bovine serum albumin for 1 h, then washed with TBST three times, added with GAGE12I antibody (1 : 100), or GAPDH antibody (1 : 100) as a loading control, left at 4°C overnight, washed with TBST three times, and then incubated with the secondary antibody for 1 h. After being washed with TBST, the ECL chemiluminescent substrate reagent kit (Thermo Fisher, USA) was used for luminescence and the image was taken by gel imager. The gray value of each band was analyzed, and the protein expression level was semiquantitatively analyzed using ImageJ.

### 2.8. Statistical Analysis

All the experimental data were analyzed by the SPSS21.0 software (IBM Corp., Armonk, N.Y., USA). The measurement data were expressed by (means ± SD). The statistical significance of the difference between the two groups was analyzed by the *t*-test. A 2-sided*P* < 0.05 was considered significantly different.

## 3. Results

### 3.1. Low Expression of miR-28-5p in Gastric Cancer Cells

The expression of miR-28-5p in human gastric cancer cell lines SGC-7901, AGS, and MGC-803 were significantly lower than that in normal gastric epithelial cells GES-1 (Figure 1). SGC-7901 cells with the lowest level of miR-28-5p were used for the following analyses in vitro.

### 3.2. Overexpression of miR-28-5p Inhibits Proliferation, Migration, and Invasion of Gastric Cancer Cells

SGC-7901 cells were transfected with miR-28-5p mimics or mimics control, named as miR-28-5p or miR-NC group, respectively. The results of the real-time PCR assay showed that the expression of miR-28-5p was significantly increased in a miR-28-5p group compared with that in a miR-NC group (Figure 2(a)). Moreover, the MTT assay revealed that the survival rate of SGC-7901 cells overexpressing miR-28-5p at 24 h, 48 h, and 72 h was significantly lower than that of the cells in the miR-NC group (Figure 2(b)). In addition, the migration and invasion were significantly lower in gastric cancer cells overexpressing miR-28-5p than those in cells transfected with mimics control (Figures 3(a) and 3(b)).

### 3.3. GAGE12I is a Target of miR-28-5p

Bioinformatics analysis using TargetScan and Pitar software provided the binding sites of miR-28-5p and GAGE12I, indicating that GAGE12I might be a target of miR-28-5p (Figure 4(a)). Luciferase assay was performed to validate this prediction, showing that the activity of luciferase decreased after cotransfection of miR-28-5p mimics and GAGE12I-WT (Figure 4(b)). The expression level of GAGE12I protein was significantly decreased in SGC-7901 cells after overexpression of miR-28-5p (Figures 4(c) and 4(d)).

### 3.4. Effect of GAGE12I Knockdown on Proliferation, Migration, and Invasion of Gastric Cancer Cells

After transfection of GAGE12I shRNA or shRNA control into SGC-7901cells, the expression of GAGE12I protein was effectively decreased in the shGAGE12I group compared with that in the scrambled group (Figures 5(a) and 5(b)). Furthermore, downregulation of GAGE12I significantly decreased cell proliferation (Figure 5(c)). Besides, after GAGE12I knockdown, the number of invasion and migration of gastric cancer cells were notably decreased (Figures 6(a) and 6(b)).

## 4. Discussion

MiRNAs regulate a variety of life activities in organisms and are important for cell differentiation, metabolism, and proliferation. At present, it has been found that miRNAs play regulatory roles in tumorigenesis. These miRNAs play inhibitory or promotive roles in tumor growth and metastasis [8–10]. MiRNAs do not have the function to encode proteins, but can affect life activities by regulating the expression and transcription of target gene mRNA [11]. In this study, we found that miR-28-5p can bind to GAGE12I-3′-UTR, and negatively regulate the expression of GAGE12I, indicating that GAGE12I is the target gene of miR-28-5p.

miR-28-5p is currently found to be closely related to tumor progression and is downregulated in liver cancer and B-cell lymphoma studies, which have shown that miR-28-5p may be a tumor suppressor [12, 13]. Studies in gastric cancer suggested that the expression of miR-28-5p is decreased in gastric cancer tissues, and the expression level of miR-28-5p is closely related to tumor metastasis and invasion [14]. The results of this study showed that the expression of miR-28-5p in gastric cancer cells was significantly lower than that in normal gastric epithelial cells, indicating that the expression of miR-28-5p in gastric cancer was downregulated, which was consistent with the above results [14]. This study also confirmed that overexpression of miR-28-5p could inhibit the proliferation, migration, and invasion of gastric cancer cells, indicating the potential therapeutic value of miR-28-5p in cancers. We hypothesized that might be associated with the cell cycle process, apoptosis, and epithelial-mesenchymal transition, which should be explored in the future. The function of miRNA is achieved by regulating its target expression. This study first suggested GAGE12I as a target of miR-28-5p in gastric cancer cells, which was confirmed by luciferase activity assay.

GAGE12I is a member of the GAGE family. With the increase of the metastatic potential of gastric cancer, the expression level of GAGE12I is gradually elevated [5, 15–17]. At present, there are few studies on GAGE12I. GAGE family genes are related to the prognosis of ovarian cancer and are also involved in the chemotherapy tolerance of ovarian cancer. GAGE7 plays an antiapoptosis role in cervical cancer. GAGE12B can promote the metastasis and growth of gastric cancer cells [18–22]. We found that the downregulation of GAGE12I could inhibit the invasion and migration of gastric cancer cells and decrease the proliferation of gastric cancer cells, indicating that GAGE12I is a promoter of gastric cancer progression. We also demonstrated that miR-28-5p regulated gastric cancer progression by targeting GAGE12I. To better understand, the role and mechanism of miR-28-5p in gastric cancer, in vivo experiments in more complicated conditions should be performed in the future [23–27].

In summary, the expression of miR-28-5p is downregulated in gastric cancer cells. Overexpression of miR-28-5p can suppress the proliferation, invasion, and migration of gastric cancer cells. The regulation of gastric cancer cell progression by miR-28-5p is related to the targeting of the GAGE12I gene, which is important for the study of the mechanism of gastric cancer genesis and metastasis.

## Figures and Tables

**Figure 1:** Low expression of miR-28-5p in gastric cancer cells. Note: compared with GES-1, ^*∗*^*P* < 0.05.

**Figure 2:** Overexpression of miR-28-5p inhibits proliferation of gastric cancer cells. (a) Overexpression of miR-28-5p in SGC-7901 cells; compared with miR-NC, ^*∗*^*P* < 0.05. (b) Overexpression of miR-28-5p inhibited the proliferation of SGC-7901 cells. Compared with miR-NC, ^*∗*^*P* < 0.05.

**Figure 3:** Overexpression of miR-28-5p inhibits invasion and migration of gastric cancer cells. (a) Cell migration test, ^*∗*^*P* < 0.05 compared with miR-NC. (b) Cell invasion test; compared with miR-NC, ^*∗*^*P* < 0.05.

**Figure 4:** miR-28-5p targets GAGE12I. (a) The 3′UTR of GAGE12I contains a nucleotide sequence complementary to miR-28-5p. (b) Luciferase reporter gene test; compared with miR-NC, ^*∗*^*P* < 0.05. (c) Western blot was used to determine the expression of GAGE12I protein in gastric cancer cells after overexpression of miR-28-5p. (d) GAGE12I protein expression. Compared with miR-NC, ^*∗*^*P* < 0.05.

**Figure 5:** Knockdown GAGE12I inhibits the proliferation of gastric cancer cells. (a) Western blot was used to determine the knockdown effect. (b) GAGE12I protein expression; compared with scrambled, ^*∗*^*P* < 0.05. (c) Knocking down GAGE12I on the survival rate of gastric cancer cells. Compared with scrambled, ^*∗*^*P* < 0.05.

**Figure 6:** Knockdown GAGE12I inhibits invasion and migration of gastric cancer cells. (a) Knocking down GAGE12I on gastric cancer cell migration; compared with scrambled, ^*∗*^*P* < 0.05. (b) Knockdown of GAGE12I on gastric cancer cell invasion. Compared with scrambled, ^*∗*^*P* < 0.05.

## Data Availability

The data used to support the findings of this study are available from the corresponding author upon request.
